# Environmental Affection-Driven English Tense Analysis: A Healthcare Exercise-Based Corpus Case Study over Public English Environment

**DOI:** 10.1155/2022/9497554

**Published:** 2022-06-11

**Authors:** Yiling Ding, Tianhua Wang

**Affiliations:** ^1^Heilongjiang University, Harbin 150080, China; ^2^Harbin Normal University, Harbin 150080, China

## Abstract

Most international academic papers are written in English, and the use of tenses in English academic papers often follows some conventional rules. Automatically extracting and analyzing English tenses in scientific papers have begun to attract researchers' attention for the global environment. In the analysis of the English tense of scientific papers, consider that the neural network model that combines attention mechanism and sequential input network such as Long Short-Term Memory (LSTM) network has a long training time, low extraction accuracy, and cannot parallelize text input. We propose an environmental affection-driven English tense analysis model, which includes an attention mechanism and LSTM model and conducts a temporal analysis of English texts based on an affective computing model. In this paper, our proposed method is verified based on the self-built healthcare exercise-based corpus over public English environment. By comparison, the experimental results show that the method proposed in this paper has better performance than ordinary Convolutional Neural Network (CNN), Support Vector Machine (SVM), and LSTM based on attention mechanism.

## 1. Introduction

English tense (tense) is a verb form that expresses behavior, action, and state under various time conditions. It is a very basic and important grammar knowledge. Different tenses are used to express different times and ways of verbs. According to traditional grammar, there are 16 tenses in English. Specifically, there are four kinds of time: present, past, future, and past and future. There are also four kinds of action: general, ongoing, complete, and complete, and the combination of time and action will produce 16 tenses. English tenses involve every complete sentence and are widely and universally used. After comparing the expression forms of English and Chinese tenses, it is not difficult to find that English tenses are mostly reflected in grammatical forms, while Chinese use more function words or combinations of other words to express the concept of tenses, lacking grammatical morphological changes, which makes English learners in China, including scientific and technological workers, have constant difficulties in the process of tense acquisition, learning and use, which is undoubtedly a great challenge for a new language knowledge [1, 2]. Most of the international academic papers are written in English. For the vast number of Chinese research paper researchers, the tense of English papers is both the key and the difficulty.

In recent years, researchers have introduced machine-learning methods into the fields of English tense analysis, English semantic understanding, multilingual tense conversion, and English-Chinese translation. However, these methods all belong to the category of shallow learning, and the function models and calculation methods are relatively simple, which makes them unable to express some complex functions with positive samples and calculation units, and the general ability is weak. At the same time, a large number of data features need to be manually selected. These defects have caused machine-learning methods to encounter bottlenecks in this task. Deep learning can automatically learn important feature representations from raw data to handle various complex tasks and has obvious advantages in modeling, interpretation and expression capabilities, and optimization. Convolutional neural network (CNN) [3, 4] and recurrent neural expressive ability and optimization have obvious advantages. CNNs can extract localized structural information in data, while recurrent neural networks [5] can process serialized structural information. In recent years, there has also been a composite model combining the two model structures, which has achieved friendship effects in the field of English tense analysis. The attention mechanism is the latest achievement in the current deep learning field, which can capture the most representative features in the text and optimize the model structure [6–8].

Sentiment analysis, also known as opinion mining, refers to people's sentiments, opinions, evaluations, attitudes, and affections about services, products, organizations, individuals, issues, events, topics, and their attributes. Text sentiment analysis is a branch of sentiment analysis, whose purpose is to judge the speaker's sentiment toward things from the original text. Machine learning based methods can be applied in the field of sentiment analysis. The tendency calculation of text sentiment is helpful for the tense understanding and verification of scientific papers. Using environmental affection-driven analysis of English tenses in scientific papers can better understand and judge the accuracy of tense use. This paper considers including environmental affection analysis into English tense analysis, analyzes English tense based on environmental affection drive, proposes an English tense analysis method based on environmental affection drive, and evaluates it using a corpus based on healthcare exercise.

The main contributions of our paper can be summarized as follows: (1) An environmental affection-driven English tense analysis method is proposed, and the affective computing model is integrated into the English tense analysis framework to improve the system performance. (2) An attention mechanism is introduced, which can give more consideration to contextual temporal correlation, and the attention mechanism is integrated with the LSTM model to analyze the English tense. (3) The method proposed in this paper is compared with three types of popular methods, from the perspective of system performance and operating efficiency. The effectiveness of this method was evaluated.

This paper is organized as follows: Section 2 describes the related work.  Section 3 details our method.  Section 4 provides the evaluation results of our method.  Section 5 concludes our paper at last.

## 2. Related Work

Murata [9, 10] used various machine-learning methods (K-proximity algorithm, decision table, maximum entropy, support vector machine) to deal with Japanese-English tense translation and found that support vector machine works best. Gong et al. [11] proposed an N-gram-based temporal translation model and synthesized it with a phrase-based statistical machine translation system. In this model, the tense of a certain verb in an English sentence is called intra-sentence tense, and the tense of a verb in the main clause of an English sentence is called inter tense. The respective N-gram models are trained by constructing an intra-sentence temporal sequence corpus and an inter-sentence temporal sequence corpus. Then, using these two N-gram models to correct the probability value of the translation result, the BLEU value increased from 28.30 to 28.92. However, the model does not utilize the information of temporal words, temporal adverbs, and temporal particles of Chinese sentences, and only uses the tense N-gram model to guess the possible temporal sequences.

In recent years, deep learning technology has made significant breakthroughs in text classification tasks, and many scholars have used deep learning technology to solve specific target sentiment analysis problems. Nguyen and Shirai [12] proposed a target-specific sentiment analysis model based on RNN and dependency tree. Dong et al. [13] proposed an adaptive RNN for the target-specific Twitter text sentiment classification task. These methods use deep learning technology to solve the problem of specific target sentiment analysis, which can better learn the sentiment feature information of text through deep neural network without the need for sentiment dictionary, and achieve better classification results than traditional machine learning methods. However, these methods need to use external knowledge such as dependency tree and syntactic relationship, and the network model structure is relatively complex. Ruder et al. [14] proposed a hierarchical bidirectional LSTM network for target-specific sentiment analysis. This method uses a bidirectional LSTM network to extract and learn features from the input text at different levels, which can effectively learn the internal relationship of sentences and the relationship between sentences. Therefore, the affective polarity of a specific target can be judged. However, the main disadvantage of the deep learning based methods is that they cost too much time on training. This limits the application. In this paper, we introduce an environmental affective computing model and combine it with the deep learning technology to analyze the English tense.

## 3. Our Method

The topological relationship between words is crucial for text temporal analysis, and language models based on recurrent neural network (RNN) are more suitable for processing text sequence data. RNN consists of three modules, namely input layer, hidden layer, and output layer [15, 16]. In the RNN model, the temporal input layer and the temporal hidden layer are aggregated into a new input layer, which also serves as the hidden layer at time *t*. The recurrent structure of RNN enables the hidden layer to retain all the information in the previous words to improve the ability to recognize the sequential relationship between words [17, 18]. There are too many unrolled state layers in the back-propagation of the RNN model through the Temporal Optimization Algorithm (BPTT), which causes the gradient of historical information to decay during training [19]. In this paper, LSTM is used to avoid the long-term dependence of the model on words, and its structure is shown in Figure 1. RNN with LSTM can be seen as an improved model of traditional RNN language model, which takes text sentences as input sequence to calculate the error of each model. But when the text sequence information is long, the RNN model with LSTM can effectively overcome the problem of sequence information decay [20]. Compared with traditional RNN language models, RNN with LSTM can fully cover longer sentences, and it performs well in multiple validation experiments, especially for English sentence structures with connectives.

The environmental affection-driven LSTM proposed in this paper introduces an attention mechanism and an environmental affection-driven computational model to improve performance, and the overall architecture is shown in Figure 1. There are six steps included in total, which are the following: environmental affection-driven computational model establishment, LSTM construction, attention mechanism inclusion, natural language inference instantiation, pooling and feature fusion, model training, and testing.

### 3.1. Environmental Affection-Driven Computational Models

The propensity calculation of text sentiment [21, 22] is helpful for the temporal understanding and verification of scientific papers. In this paper, a sentiment-driven computational classification model S_EPD_ is established, namely: *S*_EPD_ = {*E*, *P*, *D*, *C*, *G*}. In the formula, *E* is the affective tendency set; *P* is the temporal affective feature set; *D* is the affective feature degree score set; *C*: *D* ⟶ *P* is a surjective function; *G*: *C* ⟶ *E* is also a surjective function.

*E* is the set of affective tendencies of scientific papers, and if affections are divided into *m* categories, then *E* = {*e*_1_, *e*_2_,…, *e*_m_}. P is a set of temporal affective features, and if there are *n* features, then *P* = {*p*_1_, *p*_2_,…, *p*_n_}. *D* is the set of degree scores of a sentence in the paper on each affective feature, namely *D* = {*d*_1_, *d*_2_,…, *d*_n_}. When *k* degree words d_w appear in the feature *p*_i_ in a sentence, then *d*_*i*_=∏_*j*=1_^*k*^*d*_*w*_*j*_.

*C*: *D* ⟶ *P* is a surjective function connecting sentiment degree to feature, that is, *C*(*P*) = *d*_*i*_*p*_*i*._*G*: *C* ⟶ *E* is a surjective function connected by the degree of modified affection-to-affection inclination. The category of the final affective tendency is determined by the Softmax function:

(1) $$\begin{array}{c} \begin{array}{c} f_{i}\left(E\right)=\frac{e^{E_{j}}}{\sum_{l=1}^{J}e^{E_{l}}}E \end{array}. \end{array}$$

### 3.2. LSTM Construction

The LSTM model is used to deal with the problem of sequence labeling, which can make full use of the information of the entire text sequence, including the relationship information between each word, and use this information for the processing of each word [23, 24]. An LSTM model contains many LSTM cells, each LSTM cell contains an input gate, an output gate, a forget gate, and a memory cell [25, 26]. Let *c* represent the memory unit of the LSTM model, *x* the input gate of the LSTM model, *f* the forgetting gate of the LSTM model, and *h* the output gate of the LSTM model. Take the text local features {*x*_1_, *x*_2_,…, *x*_m_} as input, take the t_th_ word as an example, activate the memory unit, and obtain the feature value of each state of the t_th_ LSTM unit. The word is as follows:

(2) $$\begin{array}{c} {\tilde{F}}_{c_{t}}=\text{rec}\left(W_{xc}X_{t}+W_{hc}F_{h_{t-1}}+b_{c}\right), \end{array}$$

(3) $$\begin{array}{c} F_{i_{t}}=\sigma \left(W_{xi}X_{t}+W_{hi}F_{h_{t-1}}+W_{ci}F_{c_{t-1}}+b_{i}\right), \end{array}$$

(4) $$\begin{array}{c} F_{f_{t}}=\sigma \left(W_{xf}X_{t}+W_{hf}F_{h_{t-1}}+W_{cf}F_{c_{t-1}}+b_{f}\right), \end{array}$$

(5) $$\begin{array}{c} F_{c_{t}}=F_{f_{t}}⊙F_{c_{t-1}}+F_{i_{t}}⊙{\tilde{F}}_{c_{t}}, \end{array}$$

(6) $$\begin{array}{c} \begin{array}{c} F_{o_{t}}=\sigma \left(W_{xo}X_{t}+W_{ho}F_{h_{t-1}}+W_{co}F_{c_{t-1}}+b_{o}\right) \end{array}, \end{array}$$

(7) $$\begin{array}{c} F_{h_{t}}=F_{o_{t}}⊙\;\tan\;h\left(F_{c_{t}}\right). \end{array}$$

Among them, rec is the activation function; *W* represents the weight matrix of LSTM; *b* represents the bias vector of LSTM; *σ* is the sigmoid function; ⊙ represents the pointwise product. Similarly, after building the reverse LSTM model, the output feature of each word of the bidirectional LSTM contains the information of the entire sentence.

### 3.3. Attention Mechanism Inclusion

The attention probability is calculated using the attention mechanism [27, 28]. Attention probability can highlight the importance of a specific word to the whole sentence, and the introduction of attention mechanism considers more contextual temporal associations [29]. Therefore, the model needs to evaluate the importance of the information generated at different moments, thus introducing the attention mechanism.

In this paper, the state of each moment of the hidden layer output by the third layer is taken as the hidden state set *A* = (*a*_*M*_^1^, *a*_*M*_^2^,…, *a*_*M*_^*t*^), where *a*_*M*_^*T*^ represents the state of hidden layer of the last layer of LSTM at the t_th_ moment, and using A as the input of the attention mechanism. We can calculate the degree *e*_*t*_^*t*′^ that the output sequence at time *t* needs to pay attention to the hidden state at time *t*′. *e*_*t*_^*t*′^ can be calculated by building a simple neural network, the network parameters are *W*_h_ and *b*_h_, as shown in the following formula:

(8) $$\begin{array}{c} \begin{array}{c} e_{t}^{t^{\prime }}=\tanh\left(W_{h}\left[a_{M}^{t-1},a_{M}^{t^{\prime }}\right]+b_{h}\right) \end{array}. \end{array}$$

After obtaining *e*_*t*_^*t*′^, the weight *α*_*t*_^*t*′^ of which the output sequence at time *t* pay attention to hidden state at time *t*′ can be calculated, as shown in the following formula. That is to find the proportion of the attention degree at time t' to the attention degree at all times.

(9) $$\begin{array}{c} \begin{array}{c} \alpha_{t}^{t\prime }=\frac{\exp\left(e_{t}^{t\prime }\right)}{\sum \exp\left(e_{t}^{t\prime }\right)} \end{array}. \end{array}$$

Therefore, the total weight factor *r*_t_ at time *t* is obtained as follows:

(10) $$\begin{array}{c} r_{t}=\sum \alpha_{t}^{t\prime }a_{M}^{t\prime }. \end{array}$$

The final output of LSTM at time *t* is obtained as follows:

(11) $$\begin{array}{c} \begin{array}{c} y_{t}=\text{LSTM}\left(r_{t},a_{t-1},c_{t-1}\right) \end{array}. \end{array}$$

### 3.4. Natural Language Inference Instantiation

The purpose of natural language inference (NLI) is to establish the semantic relationship between the premise sentence and the corresponding hypothesis sentence. A total of 32 sentences and their corresponding passive voice sentences are syntactically annotated. Following Bowman's standard procedure, two sentence encoding models are introduced in this paper, with binding parameters for premise sentences and hypothetical sentences respectively. Given the output codes *s*^*p*^ and *s*^*h*^ of the hypothetical premise, the relationship can be expressed as the concatenation of *s*^*p*^, *s*^*h*^, *s*^*p*^−*s*^*h*^ and *s*^*p*^ ⇔ *s*^*h*^. This is fed into a 300D fully connected layer, which is then fed back into the three-unit output layer and Softmax for computing the probability distribution of the model's three relationships.

### 3.5. Pooling and Feature Fusion

Pooling is to perform statistical calculation on the output results of the model, and use the maximum pooling method to pool the corresponding output features *F* = {*F*_1_, *F*_2_,…, *F*_*m*_} after the attention mechanism is introduced to the entire sentence.

(12) $$\begin{array}{c} d=\text{Maximize}\left(F\right). \end{array}$$

After pooling, the overall feature *d* of the text is obtained. Regardless of the length of the sentence, the feature dimension after pooling is fixed, which solves the problem of different lengths of text sentences.

Feature fusion is to fuse multiple features into one feature, which can achieve the effect of complementary advantages of multiple features. The local features of the text and the overall features of the text are fused to obtain a new feature *F*′; then the fused feature *F*′ is imported into the classifier for relation classification, and the classification result *s*(*x*) is output.

### 3.6. Model Training and Testing

Similar to supervised machine learning methods, the dataset is divided into training data and test data. The model is then trained using the training data to learn the relevant parameters of the network. The relation classification problem is regarded as a multiclassification problem judgment. In order to obtain the optimal model, this paper conducts model training by minimizing the negative log-likelihood function. Assuming that the relationship label type *μ*∈T obtained from the target relationship is *s*(*x*) after being processed by the classifier, *T* represents the relationship label, and is converted into a conditional probability after being processed by the classifier. The probability that the label type of the target relation *y* is *μ* is

(13) $$\begin{array}{c} \begin{array}{c} p\left(y=\frac{\mu }{s\left(x\right)},\theta \right)=\frac{\exp\;{\left(s_{\theta }\left(x\right)\right)}_{\mu }}{\sum \exp\;{\left(s_{\theta }\left(x\right)\right)}_{i}} \end{array}. \end{array}$$

The stochastic gradient descent algorithm is used to minimize the negative log-likelihood function, and the objective function *J*(*θ*) of the model optimization is calculated as follows:

(14) $$\begin{array}{c} J\left(\theta \right)=-\sum_{i=1}^{D}\log\left(p\left(y=\frac{y_{i}}{x_{i}},\theta \right)\right). \end{array}$$

Among them, *θ* *=* (*W*, *U*, *V*) represents the model trainable parameters; D represents the number of training samples; (*x*_i_, *y*_i_) represents that the relationship label corresponding to the i_th_ sample *x*_i_ in the training sample is *y*_i_. Next, test data is fed into the model to evaluate performance. Because of the limited size of the dataset, validation data is not used here. Meanwhile, since the system considers language-independent annotation schemes, K-fold validation can be used to improve the performance of the dataset.

## 4. Experimental Evaluation

### 4.1. Healthcare Exercise-Based Corpus

The method proposed in this paper requires an annotated language dataset, and in order to train, develop, train, and evaluate the system, a self-built healthcare exercise-based corpus case study is used. A corpus refers to a collection of corpus of a certain size that is specially collected for one or more applications, has a certain structure, and can be retrieved by a computer program [30]. The structural and representative characteristics of a corpus are often determined by the category information under the corpus. More specifically, the distribution of categories completely determines the characteristics of the corpus.

The self-built corpus in this paper mainly includes self-built book-type literature and self-built journal type literature. The author selects all medical and health papers from the SCI (American Science Citation Index) database, because the SCI database is the most widely used and highly recognized database in the world. It has good retrieval quality and includes a high level of journal. In China, the quantity and quality of papers included in SCI are also used as important indicators to evaluate the level of scientific research. In this paper, a total of 112 medical and health related scientific papers in nine categories are selected from more than a dozen international authoritative journals as research samples. The specific distribution is shown in Figure 2. Each circle represents a category of medical and health scientific research papers, which are the following: COVID-19 (16), Depression (15), Mental Health (15), Dementia (14), Epidemiology (14), Metabolic Syndrome (13), Diabetes (9), Oral Health (8), Obesity (8). The number of papers is in brackets. Each scientific paper can be divided into six parts, namely: Abstract, Introduction, Related Work, Model and Approach, Experimental Results, Conclusion.

### 4.2. Evaluation Metrics

In this paper, three metrics which are *precision, recall,* and *F-score*, are used for evaluating model performance. They are calculated as follows:

(15) $$\begin{array}{c} \text{Precision}=\frac{TP}{TP+FP}, \end{array}$$

(16) $$\begin{array}{c} \text{Recall}=\frac{TP}{TP+FN}, \end{array}$$

(17) $$\begin{array}{c} F1-\text{score}=\frac{2\cdot \text{Precision}\cdot \text{Recall}}{\text{Precision}+\text{Recall}}. \end{array}$$

Among them, TP is the number of correctly predicted samples as positive, FP is the number of wrongly predicted samples as positive (they are negative samples actually), and FN is the number of wrongly predicted samples as negative (they are positive samples actually).

### 4.3. Parameter Setting

The activation function of the model uses the rectified linear activation (ReLU) function, the number of hidden layer nodes is 300, and softmax is used as the classifier. In order to prevent the overfitting phenomenon in the model calculation process, the L2 regularization method is used to constrain the network parameters, and the dropout strategy is also introduced in the training process, and the dropout rate is set to 0.5. In addition, the batch Adadelta optimization method is used for model training, the batch size is taken as 50 (Refer to citation [31]), and the number of training rounds is taken as 500. Among them, the code loss rate and the number of training rounds are both obtained by fivefold cross-validation, and the validation set is randomly obtained from the training samples.

### 4.4. Experimental Results

The method proposed in this paper is compared with the following three types of methods:

1. *CNN*. Based on the convolutional neural network model proposed in the literature [32], it is the most basic convolutional neural network.
2. *SVM*. The feature-based SVM classification model proposed in literature [33] achieves better classification results than previous studies.
3. *AT-LSTM*. The LSTM network based on attention mechanism proposed by the literature [34], and this model achieves better classification effect than the traditional LSTM network in the sentiment classification of five specific targets.

The experiments are carried out on our self-built healthcare exercise based corpus to analyze the performance of the proposed method. The experimental results are shown in Tables 1–3.

We first compare the accuracy, recall, and *F*-value of four different methods on our self-built corpus. The horizontal axis corresponds to the different categories of the healthcare exercise corpus. It can be seen that the method proposed in this paper is better than the other three methods in terms of precision, recall, and F1 value. The performance of AT-LSTM is second, and the performance of CNN and SVM is similar, ranking last. At the same time, it can be seen from the tables that on different types of medical and health corpora, the performance of various methods is similar, and only fluctuates within the normal range.

Next, we compare the operating efficiency of the method proposed in this paper with CNN, SVM, and AT-LSTM. The experimental results are shown in Figures 3-4, where the vertical axis represents the training time, the unit is in seconds.  Figure 3 only shows the operating efficiency of the method proposed in this paper in different categories of medical and health corpora. It can be seen that the training time of different categories is similar, and there is no obvious difference.

The horizontal axis of Figure 4 represents the number of words. It can be seen from the experimental results that in general, the method proposed in this paper does not have an advantage in terms of training time, and its training time is slightly lower than that of AT-LSTM, but much higher than that of CNN and SVM. As the number of words increases, the training time will gradually increase. Considering that the training process can be carried out offline or implemented by a higher-performance computer, although the method proposed in this paper is much less efficient in training than CNN and SVM, from the perspective of performance advantages, the method in this paper is still significant. Better than the other three methods.

## 5. Conclusion

For the tense of English verbs, “time” includes “present,” “past,” “future,” and “past future,” “tense” includes “general,” “perfect,” “perform,” and “perfect progression.” There are 16 tenses in total. Most of the international academic papers are written in English. For the vast number of Chinese research paper researchers, the tense of English papers is both the key and the difficulty. Scientific papers can generally be divided into six parts: Abstract, Introduction, Related Work, Model and Approach, Experimental Results, and Conclusion, and their writing generally has a rigorous, objective, and refined scientific style. From a microscopic point of view, scientific papers must also present some regular language features, including tense, voice, and personal usage. In order to automatically extract and analyze English tenses in scientific and technological papers, this paper designs an English tense analysis based on environmental affection-driven analysis and integrates the computational model of sentiment analysis. In order to take the contextual temporal relevance into account, this paper introduces the attention mechanism and combines the attention mechanism with LSTM to realize the temporal analysis of scientific papers. In order to verify the method proposed in this paper, this paper selects 112 medical and health related scientific and technological papers as research samples to form a corpus to carry out experiments. Compared with conventional convolutional neural network, support vector machine and LSTM based on attention mechanism, the method proposed in this paper has advantages in precision, recall, and F1-score. The experimental results show that our method is significantly better than the other three methods. In the future, the larger and more comprehensive corpus with automation technology should be considered to evaluate our method. Besides, the performance should be further improved for deployment for real cases.

## Figures and Tables

**Figure 1:** The overall framework of Our Method.

**Figure 2:** The structure of the healthcare exercise based corpus.

**Figure 3:** The training time of our method on each category of the corpus.

**Figure 4:** The training time comparison of four algorithms.

**Table 1:** The precision comparison of four algorithms.

	COVID-19	Depression	Mental health	Dementia	Epidemiology	Metabolic syndrome	Diabetes	Oral health	Obesity
Our method	88.49	89.29	90.60	90.18	91.84	92.92	93.72	92.14	90.80
AT-KSTN	85.26	84.79	85.12	86.09	84.28	85.48	84.54	83.78	86.36
CNN	82.49	83.46	82.98	81.87	80.13	79.19	77.68	76.68	77.19
SVM	77.99	76.94	77.04	79.39	81.92	83.29	78.89	78.76	78.40

**Table 2:** The recall comparison of four algorithms.

	COVID-19	Depression	Mental health	Dementia	Epidemiology	Metabolic syndrome	Diabetes	Oral health	Obesity
Our method	86.78	89.05	90.33	90.46	90.17	89.57	83.44	84.92	85.89
AT-KSTN	83.23	80.85	79.83	79.23	80.98	78.24	79.52	77.04	79.68
CNN	75.29	74.43	75.08	74.32	75.03	77.51	78.42	79.02	80.36
SVM	77.54	75.58	74.92	76.57	75.97	74.27	76.49	77.98	79.68

**Table 3:** The F1-score comparison of four algorithms.

	COVID-19	Depression	Mental health	Dementia	Epidemiology	Metabolic syndrome	Diabetes	Oral health	Obesity
Our method	87.63	89.17	90.46	90.32	91.00	91.22	88.28	88.39	88.28
AT-KSTN	84.23	82.77	82.39	82.52	82.60	81.70	81.95	80.27	82.88
CNN	78.73	78.69	78.84	77.92	77.50	78.34	78.05	77.84	78.74
SVM	77.76	76.25	75.97	77.96	78.83	78.52	77.67	78.37	79.03

## Data Availability

All data used to support the findings of the study are included within this paper.
